# MicroRNA Dysregulation in the Hippocampus of Rats with Noise-Induced Hearing Loss

**DOI:** 10.1155/2021/1377195

**Published:** 2021-09-06

**Authors:** Seungmin Ha, Kyung Woon Kim, So Min Lee, Chang Ho Lee, So Young Kim

**Affiliations:** Department of Otorhinolaryngology Head & Neck Surgery, CHA University College of Medicine, Bundang CHA Medical Center, Republic of Korea

## Abstract

Although hippocampal changes due to noise-induced hearing loss have been suggested, little is known about the miRNA levels due to these hippocampal changes. Three-week-old Sprague-Dawley rats were divided into noise and control groups (*n* = 20 per group). The noise group rats were exposed to white Gaussian noise (115 dB SPL, 4 hours per day) for three days. One day after noise exposure, the hippocampi of rats were harvested and miRNA expressions were analyzed using the Affymetrix miRNA 4.0 microarray (*n* = 6 per group). The predicted target genes of each miRNA were retrieved, and the pathways related to the predicted target genes were analyzed. miR-758-5p, miR-210-5p, miR-370-5p, miR-652-5p, miR-3544, miR-128-1-5p, miR-665, miR-188-5p, and miR-874-5p expression increased in the hippocampal tissue of the noise group compared to that in the control group. The overlapping predicted target genes included *Bend4*, *Creb1*, *Adcy6*, *Creb5*, *Kcnj9*, and *Pten*. The pathways related to these genes were the estrogen signaling pathway, vasopressin-regulated water reabsorption, thyroid hormone synthesis, aldosterone synthesis and secretion, insulin secretion, circadian entrainment, insulin resistance, cholinergic synapse, dopaminergic synapse, cGMP-PKG signaling pathway, cAMP signaling pathway, PI3K-Akt signaling pathway, TNF signaling pathway, and AMPK signaling pathway. miR-448-3p, miR204-5p, and miR-204-3p expression decreased in the hippocampal tissue of the noise group compared to that in the control group. The overlapping predicted target genes of these three miRNAs were *Rps6kas*, *Nfactc3*, *Rictor*, *Spred1*, *Cdh4*, *Cdh6*, *Dvl3*, and *Rcyt1b*. Pathway analysis suggested that the Wnt signaling pathway is related to *Dvl3* and *Nfactc3*. Noise-induced hearing loss dysregulates miR-758-5p, miR210-5p, miR370-5p, miR-652-5p, miR-3544, miR-128-1-5p, miR-665, miR-188-5p, miR-874-5p, miR-448-3p, miR-204-5p, miR-204-3p, and miR-140-5p expression in the hippocampus. These miRNAs have been predicted to be associated with hormonal, inflammatory, and synaptic pathways.

## 1. Introduction

Hearing loss affects daily life in many aspects; in particular, it hampers communication and causes psychosocial problems such as social isolation and depression [1]. One of the main causes of this handicapped condition is exposure to extreme noises [2]. Such noise exposure negatively affects hair cells in the cochlea and neurons in the auditory pathway.

Hearing loss often accompanies impaired communication skills and social isolation, which may lead to cognitive decline. The hippocampal region of the brain is involved in learning and memory, and several studies have supported the hypothesis that hearing loss induces cognitive deficit [3]. Our previous microarray study showed that acute noise exposure alters hippocampal gene expression [4]. Another study on an Alzheimer's disease (AD) model has reported that hearing loss induces cognitive deficits and reduced synapse in the hippocampus [5]. Moreover, the expression of Wnt signaling pathway molecules reduced, and amyloid-*β* and tau accumulated in the hippocampi of mice after chronic noise exposure [6].

MicroRNAs (miRNAs) are small, noncoding, single-stranded RNAs that inactivate messenger RNAs (mRNAs) [7]. miRNAs posttranscriptionally regulate gene expression almost throughout the entire human genome [8]. Since miRNAs are more stable than proteins after repeated freeze-thaw cycles, several studies have attempted to develop new biomarkers or therapeutics using miRNAs [9]. In addition, recent studies have shown a relationship between cognitive decline and miRNAs in AD. In a rat model of AD, several miRNAs were found to be involved in cognitive deficits after hearing loss [10]. Another study using aged Tg4-42 mice, a sporadic AD model revealed alterations in hippocampal miRNAs after memory decline [11].

Previous studies on miRNAs have mostly focused on chronic noise-induced hearing loss models. However, a previous study measured miRNA expression in the cochlear nucleus and inferior colliculus, not the hippocampus, after acute noise exposure [12]. Since noise-induced hearing loss and related cognitive decline may progress slowly over a long period, early diagnosis and prevention are important. Therefore, we aimed to examine the changes in hippocampal miRNAs, particularly in an early hearing loss model.

## 2. Materials and Methods

### 2.1. Animal Groups and Noise Exposure

This study was approved by the Institutional Animal Care and Use Committee of the CHA University Medical School (IACUC190046). The conditions for raising animals, noise exposure, anesthesia, and sacrifice procedures conformed to the regulations of the Institutional Animal Care and Use Committee of CHA University Medical School. Three-week-old Sprague-Dawley rats were divided into control and noise groups (Figure 1). The rats in the noise group were exposed to 2–20 kHz, 115 dB SPL noise (4 h/day for 3 days) via a free-field speaker (Tucker-Davis Technologies; Alachua, FL, USA) implemented at the top of the noise box. The noise was exposed intermittently for 3 days to attenuate stress response from continuous traumatic noise stimulation, which was lethal for some rats. Under this noise exposure schedule, hearing thresholds were not recovered over 3 months after cessation of noise exposure. The control group rats were exposed to 40–60 dB SPL background noise for 4 h/day for 3 days. All rats were not anesthetized during noise exposure. The auditory brainstem response (ABR) thresholds were measured before and after noise exposure. One day after noise exposure, all rats were euthanized and the dorsal cornu ammonis 3 region of the hippocampi was harvested [13, 14].

### 2.2. Auditory Function Tests

The ABR thresholds were measured using SmartEP (Intelligent Hearing System; Miami, FL, USA) [15] (Figure 2). The rats were anesthetized using 40 mg/kg Zoletil and 10 mg/kg xylazine. The electrodes were applied to the vertex (reference electrode), contralateral thigh (ground electrode), and ipsilateral retroauricular area (measuring electrode). The EC1 electrostatic speaker was coupled with a plastic earphone and inserted into the ipsilateral external auditory canal. Tone bursts of 4, 8, 16, and 32 kHz (duration: 1562 *μ*s, envelope: Blackman, stimulation rate: 21.1/s, amplitude: 90–20 dB SPL) were applied. The ABRs were averaged for 1024 sweeps. The lowest sound amplitude with wave III was defined as the auditory threshold.

### 2.3. Histologic Examination of the Cochlea and Hippocampus

Hematoxylin and eosin (H&E) staining and cochlear whole mount immunofluorescence were conducted for histologic examination of cochlea. Cochleae of control and noise group rats were immersion-fixed with 4% paraformaldehyde. Using 120 Mm ethylenediaminetetraacetic acid, the bony labyrinth was decalcified for 5 days. For H&E staining, the decalcified cochleae were dehydrated and embedded in paraffin. Then, 10 *μ*m sections were cut on a rotary microtome and mounted on glass slides. To examine the outer hair cells, cochlear whole mount examinations were conducted. The decalcified cochleae were dissected for the membranous labyrinth, and then, cochlear outer hair cells were identified. After washing the slides, blocking (1% Triton X-100, 1% bovine serum albumin (BSA) diluted in 10 mM PBS (pH 7.4)) and permeabilization (0.1% Triton X-100, 1% bovine serum albumin (BSA) diluted in 10 mM PBS (pH 7.4)) were performed for 1 hour at room temperature. After removing blocking solution, anti-myosin 7A (Santa Cruz, sc74516, Oregon, USA) was treated overnight at 4°C. After removing primary antibody solution, secondary antibody (Alexa 594, Abcam, ab150108, Cambridge, UK) solution (0.1% Triton X-100, 1% BSA) was incubated for 3 hours at room temperature. After removing secondary antibody solution, the tissue slides were dipped in 4′-6-diamidino-2-phenylindole dihydrochloride for 1 hour. The stained tissue slides were imaged using a confocal microscope (Zeiss LSM 880, Zeiss, Oberkochen, Land Baden-Wurttemberg, Germany).

For hippocampal histologic examination, whole brains of control and noise group rats were immersion-fixed in 4% (*v*/*v*) paraformaldehyde. The specimens were dehydrated and embedded in paraffin with optimal cutting temperature solution. For histological examination, 10 *μ*m sections were cut on a rotary microtome and mounted on glass slides. H&E staining of the hippocampus was performed to evaluate the histology of the hippocampus, especially the cornu ammonis (CA3) region. Each slide was dipped in xylene for 10 min to remove paraffin, followed by sequential washes with 100, 95, 90, 80, and 70% ethanol for 10, 10, 5, 3, and 1 min, respectively. After washing in distilled water, the sections were stained with hematoxylin for 10 min and eosin for 3 min. The stained tissue slides were imaged using an EVOSTMXL Core Imaging System (Invitrogen, Carlsbad, CA, USA, #AMEX1000). To visualize the neurons of the hippocampus, Nissl staining was performed. Briefly, deparaffinized brain sections were permeabilized and stained with NeuroTrace 530/615 Red Fluorescent Nissl (N21482, Thermo Fisher Scientific) for 20 min. After PBS washes, DAPI containing mounting solution was used for mounting. Images were photographed by using a TCS SP5II confocal microscope (Leica, Wetzlar, Germany).

### 2.4. miRNA Microarray Analyses

A total of 12 hippocampal tissues (six rats per group) were used for microarray analysis. RNA preparation and microarray analyses were conducted by BioCoRE®. The tissue was lysed using the TRIzol reagent (Life Technologies, USA). The purified RNA was quantified using a NanoDrop 1000 spectrophotometer (Thermo Scientific; Madison, WI, USA), and their quality was checked using an Agilent 2100 BioAnalyzer (Agilent Technologies; Santa Clara, CA, USA). Then, 500 ng RNA was labeled using the FlashTag Biotin RNA Labeling Kit (Affymetrix Inc.; Santa Clara, CA, USA) and hybridized using GeneChip miRNA 4.0 microarrays (Affymetrix Inc.), which contains 30,434 total mature miRNA probe sets, including 728 rat mature miRNA probe sets and 2578 human probe sets (data sheet: GeneChip miRNA 4.0 and Affymetrix miRNA 4.1 Arrays.pdf). Affymetrix miRNA arrays contain all miRNAs in miRBase Release 20. The arrays were scanned with the Affymetrix GeneChip Scanner 3000 and stored as CEL files. Raw analysis was conducted using the Transcriptome Analysis Console™ (TAC) software. CEL files were introduced into the Gene Expression Workflow in GeneSpring GX version 14.9.1 (Agilent Technologies Inc.). The RMA algorithm (background correction, log2 transformation, and probe set summarization) was implemented using default settings in GeneSpring software. Principal component analysis was performed using a covariance dispersion matrix as part of the quality control of the data. The miRNAs with ≥1.5 fold-change in expression between the noise and control group rats were considered differentially expressed. A heat map (TreeView ver.1.1.6r4) was presented for the log2 transformed differentially expressed miRNAs.

### 2.5. Confirmation of miRNA Expression Using qRT-PCR

Nine rats from each group were used for qRT-PCR analysis. Using a miScript® II RT kit (Qiagen; Hilden, Germany), 2 *μ*g RNA was mixed with reverse transcription master mix and incubated for 60 min at 37°C, after which the mixture was incubated for 5 min at 95°C and then placed on ice. A total of 20 *μ*L cDNA was diluted to 1 : 16 and used as the template cDNA. The miScript SYBR® Green PCR kit (Qiagen) was used with miScript Primer Assay reagents (Qiagen) for qRT-PCR. U6 small nuclear RNA was used as the endogenous control. The miScript Primer Assay reagents and the reaction mix were dispensed into wells containing template cDNA, sealed with a film, and centrifuged at 1000 × *g* for 1 min at room temperature. The PCR conditions were as follows: initial activation for 15 min at 95°C, followed by 40 cycles of denaturation, annealing, and extension. The fluorescence data were collected during the extension phase. The reactions were performed using an ABI 7500 real-time PCR system (Applied Biosystems; Foster City, CA, USA). Relative quantification values were obtained for each target gene using the observed cycle threshold (Ct) results and the 2^−ΔΔCt^ method.

### 2.6. The Target Gene Predictions for miRNA

The predicted target genes were retrieved for each differentially expressed miRNA using TargetScan (http://www.targetscan.org/vert_72/), and the overlapping predicted target genes were identified. The mRNA expression of predicted target genes of five or more miRNAs was explored using qRT-PCR [16, 17]. The ViiA7 real-time PCR system (Applied Biosystems; Carlsbad, CA, USA) and TOPreal™ qPCR 2× PreMIX (SYBR Green with low ROX; Enzynomics; Daejeon, Korea) were used. The primer sets used are described in Table 1. All primers were tested for amplification efficiency. Glyceraldehyde 3-phosphate dehydrogenase was used as a reference gene to normalize the amplicon levels using the 2^–ΔΔCt^ method. Then, the expression fold changes of each group were calculated and compared to those of the control group. Based on the predicted target genes confirmed using qRT-PCR, the pathways were further analyzed using DAVID Bioinformatics Resources 6.8 (https://david.ncifcrf.gov/tools.jsp).

### 2.7. Western Blotting

The protein levels of megalin, angiotensin-converting enzyme 2 (ACE2), and tumor necrosis factor *α* (TNF*α*) were measured using western blotting. The hippocampal tissue was lysed using lysis buffer (Pre-prep, Intron). The protein was purified and quantified using a microplate reader. The quantified protein samples were loaded to 8-10% sodium dodecyl sulfate-polyacrylamide gel electrophoresis. The gels were transferred to polyvinylidene difluoride membranes (Merck Millipore, Burlington, MA, USA) and incubated in blocking buffer (5% nonfat dry milk in Tris-buffered saline containing Tween-20) for 1 hour. The membranes were incubated with 1 : 1000 of anti-megalin (Santa Cruz, Dallas, Texas, U.S.A., Sc515772), anti-ACE2 (Santa Cruz, Dallas, Texas, U.S.A., Sc390851), anti-TNF*α* (Abcam, Cambridge, England, Ab6671), and anti-rabbit monoclonal *β*-actin (Cell Signaling Technology, Danvers, MA, USA, D6A8). Then, membranes were incubated with horseradish peroxidase- (HRP-) conjugated secondary antibodies (anti-rabbit IgG, HRP-linked (Cell Signaling Technology, #7074S) and goat anti-mouse IgG H&L (HRP) (Abcam, Cambridge, England, #ab97023)). Protein bands were evaluated using an enhanced chemiluminescence kit (Bio-Rad, Hercules, CA, USA) and quantified using ImageJ software (National Institutes of Health, Bethesda, MD, USA).

### 2.8. Statistical Analysis

The paired *t*-test was used to compare the ABR thresholds at pre- and postnoise exposures. The Mann-Whitney *U* test was used for analyzing the mRNA and miRNA expression levels in the noise and control group rats, after conducting the Shapiro-Wilk test. The graphs are presented as mean ± standard deviation (SD). SPSS software (ver. 21.0; IBM Corp.; Armonk, NY, USA) was used. *P* ≤ 0.05 was considered statistically significant.

## 3. Results

Auditory threshold shifts were observed at 4, 8, 16, and 32 kHz following noise exposure (Figure 2). The auditory thresholds were higher in the noise group 3 days after noise exposure than those before noise exposure (all *P* < 0.05).

Compared to the control group, the cochleae of white group rats showed loss and disorientations of outer hair cells and spiral ganglial cells (Figure 3).

Gross morphology of hippocampi was not significantly different between the control and noise groups (Figure 4). However, the noise group showed pigmented and vacuolated cells in the CA3 region which was not obvious in the control group rats.

Nine miRNAs, miR-758-5p, miR-210-5p, miR-370-5p, miR-652-5p, miR-3544, miR-128-1-5p, miR-665, miR-188-5p, and miR-874-5p, were upregulated in the hippocampal tissue of noise group rats (Table 2), which was confirmed using qRT-PCR. miR-758-5p was the most upregulated, with 2.23-fold (SD = 0.14) higher expression in noise-induced rats than in normal rats.

The overlapping predicted target genes of five or more upregulated miRNAs were selected. qRT-PCR results demonstrated that *Bend4*, *Creb1*, *Adcy6*, *Creb5*, *Kcnj9*, and *Pten* were downregulated in the hippocampal tissues of the noise group rats (Figure 5).

The mRNA expression levels of *Bend4*, *Creb1*, *Adcy6*, *Creb5*, *Kcnj9*, and *Pten* were, respectively, 0.59-fold (SD = 0.10, *P* = 0.001), 0.52-fold (SD = 0.12, *P* < 0.001), 0.59-fold (SD = 0.10, *P* = 0.03), 0.20-fold (SD = 0.05, *P* < 0.001), 0.47-fold (SD = 0.10, *P* = 0.001), and 0.54-fold (SD = 0.12, *P* = 0.004) lower in the noise group rats than in the control group rats. The pathway analysis suggested that these predicted target genes were related to the estrogen signaling pathway, vasopressin-regulated water reabsorption, thyroid hormone synthesis, aldosterone synthesis and secretion, insulin secretion, circadian entrainment, insulin resistance, cholinergic synapse, dopaminergic synapse, cGMP-PKG signaling pathway, cAMP signaling pathway, PI3K-Akt signaling pathway, TNF signaling pathway, and AMPK signaling pathway (Table 3).

In protein levels, the protein expression levels of megalin, ACE2, and TNF*α* were changed in the hippocampi of noise group rats, compared to those of control group rats (Figure 6). The protein expression level of megalin was 0.72-fold lower in the noise group (SD = 0.23, *P* = 0.02). The protein expression level of ACE2 was 1.56-fold higher in the noise group (SD = 0.26, *P* = 0.004). The protein expression level of TNF*α* was 0.77-fold lower in the noise group (SD = 0.18, *P* = 0.037).

On the contrary, miR-448-3p, miR-204-5p, miR-204-3p, and miR-140-5p were downregulated in the noise group rats. Notably, qRT-PCR confirmed that miR-448-3p, miR-204-5p, and miR-204-3p were downregulated, while miR-140-5p was upregulated (1.63-fold, SD = 0.04). miR-448-3p was the most downregulated, with 0.18-fold (SD = 0.004) lower expression in noise-induced rats than in normal rats.

*Rps6kas*, *Nfactc3*, *Rictor*, *Spred1*, *Cdh4*, *Cdh6*, *Dvl3*, and *Rcyt1b* were the predicted target genes of the downregulated miRNAs (Table 2). qRT-PCR results demonstrated that these genes were upregulated in the noise group rats (Figure 7). The mRNA expression levels of *Rps6kas*, *Nfactc3*, *Rictor*, *Spred1*, *Cdh4*, *Cdh6*, *Dvl3*, and *Rcyt1b* were, respectively, 1.61-fold (SD = 0.24, *P* = 0.019), 3.20-fold (SD = 0.64, *P* = 0.002), 3.53-fold (SD = 0.63, *P* = 0.001), 1.33-fold (SD = 0.56, *P* = 0.031), 3.05-fold (SD = 0.72, *P* = 0.0008), 1.63-fold (SD = 0.20, *P* = 0.011), 1.65-fold (SD = 0.25, *P* = 0.015), and 1.86-fold (SD = 0.28, *P* = 0.005) higher in the noise group rats than in the control group rats. Pathway analysis for these upregulated genes suggested that *Dvl3* and *Nfactc3* are related to the Wnt signaling pathway.

## 4. Discussion

Noise-induced hearing loss changed the hippocampal expression levels of several miRNAs, including miR-758-5p, miR210-5p, miR370-5p, miR-652-5p, miR-3544, miR-128-1-5p, miR-665, miR-188-5p, miR-874-5p, miR-448-3p, miR-204-5p, miR-204-3p, and miR-140-5p. The predicted target genes of the upregulated miRNAs include *Creb1*, *Adcy6*, *Creb5*, *Kcnj*, and *Pten*, which are related to the estrogen signaling pathway, vasopressin-regulated water reabsorption, thyroid hormone synthesis, aldosterone synthesis and secretion, insulin secretion, circadian entrainment, insulin resistance, cholinergic synapse, dopaminergic synapse, cGMP-PKG signaling pathway, cAMP signaling pathway, PI3K-Akt signaling pathway, TNF signaling pathway, and AMPK signaling pathway. On the contrary, the predicted target genes of the downregulated miRNAs, such as miR-448-3p, miR-204-5p, and miR-204-3p, include *Rps6kas*, *Nfactc3*, *Rictor*, *Spred1*, *Cdh4*, *Cdh6*, *Dvl3*, and *Rcyt1b*, which are related to the Wnt signaling pathway. These results suggest a link between noise-induced hearing loss and hippocampal changes, which could induce cognitive dysfunction.

Hippocampal changes due to hearing loss have been suggested in noise-induced as well as in age-related hearing loss rodent models [18]. Transient threshold shift (TTS) as well as permanent threshold shift (PTS) models [19, 20] showed biochemical, neuronal, and behavioral changes in the hippocampus after noise exposure [21–23]. Within 24 h after impulse noise exposure (peak sound pressure: 165 dB SPL for 100 ms), glutamate-N-methyl-D-aspartic acid receptor (NMDAR) signaling was activated, tau hyperphosphorylation increased, and the Morris water maze test indicated diminished spatial memory [23]. The number of hippocampal neurons decreased within 2–6 h after noise exposure (4 kHz, 104 dB SPL for 30 min) [21]. The long-term potentiation of the hippocampus was inhibited after exposure to 110 dB SPL noise (12 kHz) for one minute [22]. Stress responses, including oxidative stress, inflammation, hormonal changes, and neuronal or synaptic changes related to auditory signaling deprivation, may induce hippocampal dysregulations [18]. The stress hormones, such as norepinephrine and serotonin, were elevated in the hippocampus following noise exposures [24]. In addition, inflammatory changes with dystrophic microglia and diminished neurogenesis were noted in hippocampi of noise-induced hearing loss mice [25]. The results of this study also predicted the changes in signaling pathways related to hormones, such as estrogen signaling pathway, vasopressin-regulated water reabsorption, thyroid hormone synthesis, aldosterone synthesis and secretion, insulin secretion, circadian entrainment, insulin resistance, and inflammation, such as the cGMP-PKG signaling pathway, cAMP signaling pathway, PI3K-Akt signaling pathway, TNF signaling pathway, and AMPK signaling pathway, and synaptic changes, such as cholinergic synapses and dopaminergic synapses in the hippocampi of the noise group rats. To support this, the protein expression levels of estrogen receptor protein of megalin and TNF*α* were lower in the noise group [26]. Megalin is known as a low-density lipoprotein receptor-related protein family and was suggested to have a critical role in hearing by interacting with estrogen [26]. In addition, the expression of ACE2 was higher in the noise group than in the control group in the present study. The balance between ACE and ACE2 is critical to regulate the level of angiotensin II [27]. These hippocampal changes after noise exposure could be induced by the miRNA changes following noise exposure.

Little is known about miRNA changes in the hippocampus after noise exposure. Notably, a recent study reported miRNA changes in the hippocampus of a surgically deafened AD rat model and demonstrated that miR-376a-3p and miR-598-3p expression changes in the hippocampal tissue of a rat model of amyloid-*β* infusion and bilateral cochlear ablation [10]. However, no relevant target gene or pathway was identified in the previous study. In this study, miR-758-5p, miR210-5p, miR370-5p, miR-652-5p, miR-3544, miR-128-1-5p, miR-665, miR-188-5p, and miR-874-5p expression increased in the hippocampi of the noise group rats. Among these miRNAs, miR-188-5p regulates synaptic plasticity as its expression level increases with long-term potentiation [28]. In addition, miR-188-5p diminishes amyloid-*β* peptide_1-42_-mediated synapse elimination and dysfunction and cognitive deficits by downregulating neuropilin-2 (Nrp-2) in a 5XFAD mouse model of AD [29]. *Nrp-2* is a receptor for semaphoring 3F, which plays a role in synaptic plasticity and axon guidance [30]. Thus, miR-188-5p upregulation in the hippocampal tissue of noise-induced rats may imply the induction of synaptic changes in the hippocampus after hearing loss. Moreover, miR-210-5p, which was found to be upregulated in this study, was also reported to increase in a rat model of vascular dementia [31]. miR-210-5p increase induced loss of synapses in the CA 1 region of the hippocampus in vascular dementia rats and suppressed the mRNA expression of synaptosomal-associated protein 25 [31].

In contrast, miR-448-3p, miR-204-5p, miR-204-3p, and miR-140-5p expression decreased in the hippocampi of the noise group rats in this study. miR-204-3p was downregulated in the APPswe/PS1De9 (APP/PS) mouse model of AD [32]. miR-204-3p replenishment ameliorated memory deficits and reduced oxidative stress in APP/PS1 mice by suppressing nicotinamide adenine dinucleotide phosphate oxidase 4 [32]. Although very few studies have focused on other downregulated miRNAs, the predicted target gene and pathway analyses suggested the relationship with the Wnt signaling pathway, which is involved in multiple processes involved in neurogenesis and synaptic plasticity [33].

This study explored the miRNA changes in rat hippocampi one day after noise exposure. This time frame was chosen based on previous studies reporting hippocampal changes within one day after noise exposure [21, 23]. The temporal and regional changes in miRNAs warrant further study. In addition, although several predicted target genes and pathways related to the changed miRNAs were explored, the plausible molecular networks need to be elucidated through rescue studies using these miRNAs.

## 5. Conclusions

miR-758-5p, miR210-5p, miR370-5p, miR-652-5p, miR-3544, miR-128-1-5p, miR-665, miR-188-5p, and miR-874-5p were upregulated, whereas miR-448-3p, miR-204-5p, miR-204-3p, and miR-204-3p were downregulated in the hippocampi of rats with noise-induced hearing loss. These miRNAs mediate hormonal responses, inflammation, and synaptic changes.

## Figures and Tables

**Figure 1:** The miRNA microarray in the noise-induced hearing loss rats (*n* = 20 per group). Noise was exposed for three days, and auditory threshold shifts were checked using auditory brainstem response (ABR) threshold measures. The histologic examination of cochleae and hippocampi was conducted (*n* = 2 per group). The miRNA microarray was conducted using hippocampi of the noise-induced hearing loss and control rats (*n* = 6 per group). The predicted target gene analyses were performed, and their expression levels were estimated using qRT-PCR (*n* = 9 per group). The related proteins of identified pathways were evaluated using western blotting (*n* = 3 per group).

**Figure 2:** The auditory threshold shifts after noise exposure. The auditory brainstem response (ABR) thresholds were increased after noise exposure (postnoise 3 days) compared to those before noise exposure (prenoise) at 4, 8, 16, and 32 kHz (^∗^*P* < 0.05, paired *t*-test between prenoise and postnoise 3 days; R: right side of the ear; L: left side of the ear).

**Figure 3:** Comparison of cochlear histology between control and noise group rats. (a) Hematoxylin and eosin demonstrated loss of spiral ganglion cells in the noise group rats compared to the control group. (b) Cochlear whole mount immunofluorescence showed loss and disorientation of outer hair cells in the noise group rats.

**Figure 4:** Comparison of hippocampal histology between control and noise group rats. Hematoxylin and eosin demonstrated pigmented (dotted arrows) and vacuolated (arrows) cells in the noise group rats compared to the control group. The Nissl staining of the CA3 region demonstrated neuronal cells of control and noise groups which did not show significant difference between groups.

**Figure 5:** The predicted target genes of the upregulated miRNAs in the hippocampi of noise-induced hearing loss rats. The mRNA expression levels of *Bend4*, *Creb1*, *Adcy6*, *Creb5*, *Kcnj9*, and *Pten* were lower in the noise-induced hearing loss rats than in control rats.

**Figure 6:** The protein expression levels of megalin, ACE2, and TNF*α* in the hippocampi of noise and control group rats. The protein expression levels of megalin and TNF*α* were lower, and those of ACE2 were higher in the noise group rats than in control group rats (^∗^*P* < 0.05).

**Figure 7:** The predicted target genes of the downregulated miRNAs in the hippocampi of noise-induced hearing loss rats. The mRNA expression levels of *Rps6ksa*, *Nfactc3*, *Rictor*, *Spred1*, *Cdh4*, *Cdh6*, *Dvl3*, and *Rcyt1b* were higher in the noise-induced hearing loss rats than in control rats.

**Table 1:** Oligonucleotide primer sequences for quantitative reverse transcriptase polymerase chain reaction.

Gene	Primer sequence (forward)	Primer sequence (reverse)	Annealing temperature (°C)	Product size (bp)	Sequence number
*Bend4*	5′-CTTTCTTGTTCAGCCGCCAG-3′	5′-CCCCCACCTTCCGAAAAAGA-3′	60	108	NM_020088.1
*Creb1*	5′-TCC CAC TGT AAC CTT AGT GCA G-3′	5′-ATA ACT GAT GGC TGG GCC G-3′	60	84	NM_134443.1
*Creb5*	5′-CATCTCTCGAGACCCGCTAC-3′	5′-TGGTCCTCTGTTGGGAAACG-3′	60	124	NM_001134621.1
*Adcy6*	5′-TACATGAGCTGCCTCAAGAATGT-3′	5′-GTGTGGTCACCTCAGTGTCAT-3′	60	169	NM_012821.4
*Kcnj9*	5′-AGCTGGCAGAAATGAAGAGGA-3′	5′-ACACACTCAGTCCATTGGGTT-3′	60	138	NM_017297.2
*Pten*	5′-TATCTTGTGCTCACCCTGACAAA-3′	5′-AGAAGTATCGGTTGGCCTTGT-3′	60	70	NM_031606.1
*Rps6ka5*	5′-TCCCAAGAAGCGATTGGGAT-3′	5′-CGTCCCGGATCACTGGTTTA-3′	60	83	NM_001108048.1
*Nfatc3*	5′-TAACCTCCACCCATTTGCCA-3′	5′-GACCGAAGATGGTATTATGTGCTG-3′	60	73	NM_001108447.1
*Rictor*	5′-AATACCCTGCAGCGATCCTC-3′	5′-GGAGGCACATGCTTTGACTG-3′	60	155	NM_008775080.2
*Spred1*	5′-CCCGTTCCCTGGTGAAAGAT-3′	5′-GGTATCTGGCTCACTTGGCT-3′	60	145	NM_001047089.1
*Cdh4*	5′-GCTGGTAGCCCAGACATCAT-3′	5′-TCTGGTGTTGTTGAGGCCAT-3′	60	122	NM_017602710.1
*Cdh6*	5′-GTTACAACGACGAAGGTGGC-3′	5′-TGCTGTCTCCATGGCTTAGG-3′	60	85	NM_012927.1
*Dvl3*	5′-CCTTCAATGGAACGCACAGG-3′	5′-CGTTGGGCAGATACCAAGGA-3′	60	128	NM_001107081.2
*Pcyt1b*	5′-GAGTAGCCGGATGCTACAGG-3′	5′-AGGTCTTGTTTGGGAGCCAG-3′	60	119	NM_173151.1

**Table 2:** The differentially expressed miRNAs in noise-induced hearing loss rats and their predicted target genes.

Transcript ID (miRNA name)	Regulation	Microarray		qRT-PCR			Predicted target genes							
		FC	*P* value	FC	SD	*P* value								
rno-miR-758-5p	Up	1.86	0.028	2.23	0.14	<0.001	*Bend4*	*Creb1*	*Creb5*	*Adcy6*	*Kcnj9*	*Pten*		
rno-miR-210-5p	Up	1.84	0.025	2.52	0.21	<0.001	*Bend4*	*Creb1*	*Creb5*		*Kcnj9*	*Pten*		
rno-miR-370-5p	Up	1.80	0.042	1.85	0.04	<0.001								
rno-miR-652-5p	Up	1.69	0.033	2.01	0.11	<0.001	*Bend4*	*Creb1*	*Creb5*	*Adcy6*	*Kcnj9*			
rno-miR-3544	Up	1.61	0.048	2.73	0.27	<0.001	*Bend4*	*Creb1*	*Creb5*	*Adcy6*		*Pten*		
rno-miR-128-1-5p	Up	1.61	0.048	2.29	0.08	<0.001	*Bend4*			*Adcy6*	*Kcnj9*	*Pten*		
rno-miR-665	Up	1.60	0.023	1.66	0.06	<0.001								
rno-miR-188-5p	Up	1.56	0.046	1.73	0.03	<0.001	*Bend4*					*Pten*		
rno-miR-874-5p	Up	1.53	0.022	1.9	0.04	<0.001	*Bend4*	*Creb1*	*Creb5*	*Adcy6*	*Kcnj9*			
rno-miR-448-3p	Down	0.09	0.017	0.18	0.004	<0.001	*Rps6ka5*	*Nfatc3*	*Rictor*	*Spred1*	*Cdh4*	*Cdh6*	*Dvl3*	*Rcyt1b*
rno-miR-204-5p	Down	0.16	0.015	0.35	0.01	<0.001	*Rps6ka5*	*Nfatc3*	*Rictor*	*Spred1*	*Cdh4*	*Cdh6*	*Dvl3*	*Rcyt1b*
rno-miR-204-3p	Down	0.28	0.032	0.41	0.01	<0.001	*Rps6ka5*	*Nfatc3*	*Rictor*	*Spred1*	*Cdh4*	*Cdh6*	*Dvl3*	*Rcyt1b*
rno-miR-140-5p	Down	0.58	0.043	1.63	0.04	<0.001								

**Table 3:** Pathways related to the predicted target genes of differentially expressed miRNAs in noise-induced hearing loss rats.

Term	Regulations	*P* value	Benjamini	Genes				
Estrogen signaling pathway	Down	<0.001	0.001	*Adcy6*	*Creb1*	*Creb5*	*Kcnj9*	
Vasopressin-regulated water reabsorption	Down	<0.001	0.006	*Adcy6*	*Creb1*	*Creb5*		
Thyroid hormone synthesis	Down	<0.001	0.009	*Adcy6*	*Creb1*	*Creb5*		
Aldosterone synthesis and secretion	Down	0.001	0.009	*Adcy6*	*Creb1*	*Creb5*		
Insulin secretion	Down	0.001	0.009	*Adcy6*	*Creb1*	*Creb5*		
Circadian entrainment	Down	0.001	0.009	*Adcy6*	*Creb1*		*Kcnj9*	
Insulin resistance	Down	0.001	0.009		*Creb1*	*Creb5*		*Pten*
Cholinergic synapse	Down	0.001	0.009		*Creb1*	*Creb5*	*Kcnj9*	
Dopaminergic synapse	Down	0.002	0.011		*Creb1*	*Creb5*	*Kcnj9*	
cGMP-PKG signaling pathway	Down	0.003	0.013	*Adcy6*	*Creb1*	*Creb5*		
cAMP signaling pathway	Down	0.004	0.018	*Adcy6*	*Creb1*	*Creb5*		
PI3K-Akt signaling pathway	Down	0.011	0.050		*Creb1*	*Creb5*		*Pten*
TNF signaling pathway	Down	0.055	0.170		*Creb1*	*Creb5*		
AMPK signaling pathway	Down	0.064	0.190		*Creb1*	*Creb5*		
Wnt signaling pathway	Up	0.071	1.000	*Dvl3*	*Nfatc3*			

## Data Availability

The raw data of experiments used to support the findings of this study are available from the corresponding author upon request.
